The article "Exploring Heart Rate Variability as a Biomedical Diagnostic Tool for the Disympathetic Dimension of Eight-Constitution Medicine" was published in 2021. Journal: Evid Based Complement Alternat Med.

# Exploring Heart Rate Variability as a Biomedical Diagnostic Tool for the Disympathetic Dimension of Eight-Constitution Medicine

**DOI:** 10.1155/2021/6613798

**Published:** 2021-06-15

**Authors:** Hyonna Kang, Sean Walsh, Brian Oliver, Terry Royce, Byung Je Cho

**Affiliations:** ^1^School of Life Sciences, University of Technology Sydney, Sydney, NSW, Australia; ^2^Sage Acupuncture, Sydney, NSW, Australia; ^3^Woolcock Institute of Medical Research, The University of Sydney, Sydney, NSW, Australia; ^4^Graduate Research School, University of Technology Sydney, Sydney, NSW, Australia; ^5^Chedam Hospital of Korean Medicine, Busan, Republic of Korea; ^6^Korean Medicine, Dong-Eui University, Busan, Republic of Korea

## Abstract

**Background:**

Eight-Constitution Medicine (ECM), an extension of Traditional Korean Medicine, divides the population into eight groups based on their physiological characteristics. ECM divides these eight groups into two larger groups based on autonomic reactivity: the Sympathicotonic group and the Vagotonic group (herein referred to as the Disympathetic Dimension). Heart Rate Variability (HRV) is a widely used biomedical tool to assess cardiac autonomic function. This raises the question of the utility of using HRV to correctly diagnose ECM constitutions.

**Methods:**

A systematic literature review was conducted to evaluate the correlation between HRV and constitutions in Korean Constitutional Medicine, including Eight-Constitution Medicine (ECM) and Sasang Constitution Medicine (SCM). The articles were obtained from both English (Scopus, PubMed, EMBASE, ProQuest, and Medline) and Korean databases (NDSL and RISS), in addition to Google Scholar, without date restriction. 20 studies met the inclusion criteria, and data were extracted against three aspects: (1) correlation between HRV and constitution, (2) HRV reporting and interpretation, and (3) extraneous factors that were controlled in the studies.

**Results:**

386 articles were initially identified, which was reduced to *n* = 20 studies which met the inclusion criteria. Of these, 19 were SCM studies and 1 was an ECM study. Sample sizes varied from 10 to 8498 men and women, with an age range of 10–80 years. SCM studies explored HRV differences by constitution, measuring HRV at resting, with controlled breathing, before and after acupuncture stimulation, and by other interventions. SCM studies reported either no significant differences (HRV at resting or with controlled breathing studies) or conflicting data (HRV with acupuncture stimulation studies). The single ECM study measured HRV at resting and after acupuncture stimulation but reported no significant differences between the two groups of Sympathicotonia and Vagotonia.

The article "Exploring Heart Rate Variability as a Biomedical Diagnostic Tool for the Disympathetic Dimension of Eight-Constitution Medicine" was published in 2021. Journal: Evid Based Complement Alternat Med.

**Conclusions:**

Due to inconsistencies in study design, study population, and measures of HRV, there was no consistency in the data to support the use of HRV as a biomedical determinant of ECM constitutions.

## 1. Introduction

Eight-Constitution Medicine (ECM) originates from Korean Constitutional Medicine, a further development of Sasang Constitution Medicine (SCM) [1–3]. A constitution refers to the nature of an individual's health response based on their psychosocial and physiological traits. While SCM classifies people into one of four constitutions (Tae-Yang, Tae-Eum, So-Yang, and So-Eum) [4], ECM differentiates people as one of the eight constitutions: Pulmotonia (PUL), Colonotonia (COL), Renotonia (REN), Vesicotonia (VES), Pancreotonia (PAN), Gastrotonia (GAS), Hepatonia (HEP), and Cholecystonia (CHO) (Figure 1) [5]. Consequently, ECM employs a personalized approach to treatment, even between people with the same ‘disease', prescribing individualized neuromodulatory protocols (via acupuncture) and lifestyle regimen (including dietary guidance), aligning with the emerging “personalized and preventive” medicine movement [6–8].

However, despite over 50 years of ECM research in Korea [2, 5, 9–11], differentiating a patient's constitution still primarily relies upon the practitioner's assessment of the radial arterial pulse. This requires highly developed palpatory skills to detect distinct differences in pulse position and contours that differentiate one constitution from another [12–15]. While there is greater interrater agreement reported between experienced practitioners, agreement levels, unfortunately, reduce among inexperienced practitioners [13, 14, 16, 17].

To better support reliability and remove subjectivity, a proposal is to differentiate constitutions based instead on autonomic balance. Eppinger and Hess introduced the constitutional concepts of Vagotonia and Sympathicotonia [18], which have a relationship with Heart Rate Variability (HRV). They defined Sympathicotonia as having increased tone in the sympathetic nervous system and with an abnormal increased response to adrenalin, and Vagotonia as having increased tone in the parasympathetic nervous system and with a relatively increased sensitiveness to pilocarpine [5, 18, 19]. This aligns with ECM, which proposes these hereditary factors as constitutional differences and classifies four (of the eight) constitutions into Sympathicotonic type and Vagotonic type (Figure 1) [5].

A set of biomedical diagnostics that differentiates the Sympathicotonic and Vagotonic types of ECM (referred to herein as the ‘Disympathetic Dimension') would provide objective support for assessing the eight-constitution framework. Furthermore, HRV is a widely used biomedical tool to objectively assess cardiac autonomic function [20]. While it is generally agreed that high-frequency HRV can be used to assess cardiac vagal modulation (parasympathetic) [20–25], the same cannot be said for low-frequency HRV assessing cardiac sympathetic modulation [26–31]. HRV, however, is very sensitive to a range of extraneous factors [32].

The article "Exploring Heart Rate Variability as a Biomedical Diagnostic Tool for the Disympathetic Dimension of Eight-Constitution Medicine" was published in 2021. Journal: Evid Based Complement Alternat Med.

Consequently, to explore HRV as a biomedical diagnostic for ECM, HRV studies in the Korean Constitutional Medicine (Eight-Constitution Medicine, Sasang Constitution Medicine) were critically reviewed against three considerations: (1) the correlation between HRV and constitutions, (2) HRV reporting and interpretation, and (3) controlled extraneous factors.

## 2. Methods

### 2.1. Databases

A systematic review was conducted on full-text articles obtained from both English (Scopus, PubMed, EMBASE, ProQuest, and Medline) and Korean (NDSL, RISS) electronic databases, in addition to Google Scholar, without date restriction.

### 2.2. Search Terms

Search terms for English databases include (“heart rate variability” OR HRV) AND “eight constitution”, (“heart rate variability” OR HRV) AND “8 constitution*∗*”, (“heart rate variability” OR HRV) AND “Sasang”, while Korean databases search terms include: “heart rate variability” AND 8체질, HRV AND 8체질, HRV AND 팔체질, 심박^*∗*^ AND 팔체질, 심박^*∗*^ AND 8체질, “Heart rate variability” AND 사상체질, “HRV” AND 사상체질, 심박^*∗*^ AND 사상체질.

## 3. Results

### 3.1. Review Process

From the 386 total records obtained from database search (*n* = 384) and manual searches (*n* = 2), full-text articles of *n* = 36 were obtained after excluding duplicated papers (*n* = 60) and nonrelevant papers or unavailable articles (*n* = 290). The articles (*n* = 36) were further reviewed against the inclusion criteria (i.e., short-term recordings of HRV) for Korean Constitutional Medicine (Eight Constitution or Sasang Constitution). A further 16 articles were excluded, leaving *n* = 20 papers for critical review. Of these, one was an ECM article, and the others were SCM studies (*n* = 19). The review process is presented in Figure 2.

### 3.2. Study Characteristics (Table 1)

#### 3.2.1. Demographic Characteristics

Sample sizes varied from 10 to 8498 men and women, with an age range of 10 to 80 years. 13 out of 20 studies were in healthy subjects, and the rest were either patient populations or medical information not being available.

#### 3.2.2. Study Intervention

To explore constitutional differences, the studies measured HRV at resting level [40, 43, 45, 53] with paced breathing [34, 36, 54], after acupuncture stimulation [38, 39, 41, 44, 47, 51, 52], or other interventions such as meditation [37], forest healing program [42], autogenic training [48], emotional stimulus [50], and constitutional herbal formula [46].

The article "Exploring Heart Rate Variability as a Biomedical Diagnostic Tool for the Disympathetic Dimension of Eight-Constitution Medicine" was published in 2021. Journal: Evid Based Complement Alternat Med.

#### 3.2.3. HRV Analysis and Devices

HRV analysis studies varied: time and frequency domain (*n* = 15), frequency domain only (*n* = 4), and time domain only (*n* = 1). All studies used commercial HRV medical devices of ECG (*n* = 16), PPG (*n* = 2), or IBI (*n* = 2).

### 3.3. Correlation between HRV and Constitution

#### 3.3.1. ECM and HRV at Resting and after Acupuncture Stimulation (*p* < 0.05) (Table 2)

A single ECM study [33] measured HRV baseline at resting and after constitutional acupuncture (i.e., a predefined acupuncture formula for a specific constitution) stimulation but reported no significant differences between the two groups of Sympathicotonia and Vagotonia. The study had a small sample size (42 patients), wide age range (14–73 yr), uncontrolled gender factors, and a short observation period after acupuncture.

#### 3.3.2. SCM and HRV at Resting (*p* < 0.05) (Table 3)

None of the SCM studies reported significant differences in HF at resting between constitutions. Two relatively well-controlled SCM studies indicated Tae-Eum constitution (with characteristics of increased parasympathetic reactivity) showed a lower LF/HF ratio than the So-Yang constitution (with both parasympathetic and sympathetic reactivity) at resting condition (*p* < 0.05) [43, 47, 55].

#### 3.3.3. SCM and HRV with Controlled Breathing (*p* < 0.05) (Table 4)

Three SCM studies explored the effects of different breathing approaches on constitutions by measuring HRV: breath-counting meditation [36], paced breathing (3, 6, or 12 times per min) [34], and the ratio of inhalation and exhalation (4 : 6 and 6 : 4, respectively) with posture changes [35], but HRV measures from both baseline and controlled breathing showed no difference between constitutions.

#### 3.3.4. SCM and HRV after Acupuncture Stimulation (*p* < 0.05) (Table 2)

5 out of 7 SCM acupuncture studies reported some HRV differences between constitutions. Two within-subject studies [38,41] reported that Taegeuk acupuncture stimulation (i.e., a predefined acupuncture formula for a specific constitution) resulted in a significant increase in HFnu in both the Tae-Eum and So-Yang type compared to a resting or stress condition, indicating a relative increase in cardiac vagal modulation. Three between-subject studies based on different acupuncture stimulation methods reported different HRV measures or conflicting data: (1) So-Yang type showed higher SDNN than So-Eum type and Tae-Eum type during passive coping conditions (i.e., enduring pain passively) and the opposite during active coping condition (i.e., pain stimulation will stop when signaling) when pain is induced by electroacupuncture [51]; (2) So-Eum type showed higher rMSSD compared to Tae-Eum type and Tae-Eum type showed higher LFnu and LF/HF compared to So-Eum type based on changes between right after needle insertion at LR3 and LI4 and 1 hour after needle removal [52]; (3) LFnu and LF/HF were increased in So-Yang type and LF/HF was significantly higher in So-Eum type compared to So-Yang type, while LF/HF of Tae-Eum type was in between, after acupuncture stimulation at LI4 only [47].

The article "Exploring Heart Rate Variability as a Biomedical Diagnostic Tool for the Disympathetic Dimension of Eight-Constitution Medicine" was published in 2021. Journal: Evid Based Complement Alternat Med.

#### 3.3.5. SCM and HRV after Other Interventions (*p* < 0.05) (Table 5)

So-Eum type had significantly enhanced HRV (i.e., SDNN) after either a meditation program [37] or an autogenic training program [48]. SDNN (time domain variable) results recorded on short-term HRV, however, may need further validation of reproducibility.

### 3.4. HRV Reporting and Interpretation

#### 3.4.1. Reporting of HRV Measures (Table 6)

The number of reported HRV variables varied from more than five (*n* = 9) to only one (e.g., SDNN or LF/HF) (*n* = 2). The most frequently reported variable was SDNN (*n* = 16), and the least was mRR (*n* = 4). Frequency domain variables were used to describe sympathovagal modulation: LF/HF (*n* = 14), LF and HF power (*n* = 12), LFnu and HFnu (*n* = 11), and natural logarithm (*n* = 3). Other HRV influencing parameters reported include mean heart rate (*n* = 13), respiration rate (*n* = 1), and blood pressure (*n* = 3).

#### 3.4.2. Normalized Units and Raw Values (Table 7)

13 of the 20 studies reported multiple nu/ratios (i.e., HFnu, LFnu, and LF/HF ratio), and this could present potential problems of redundancy and interpretation, especially when the HRV reporting measures provide inconsistent outcomes, as noted in Heathers' HRV methodology study [32]: for example, if LFnu was significant and LF/HF not, this might be interpreted as a change in sympathetic activity but there is no sympathovagal balance. Some SCM and HRV studies reported redundant [43] or inconsistent results: for example, LFnu increased in So-Yang type, but there is no change in HFnu [47], or HFnu was higher in So-Yang type than Tae-Eum type but there is no difference in LHnu [52]. While the task force recommended that research should always report both raw values and normalized units [56] because the changes in the individual frequency bands may be inconsistent with the reporting of lone normalized HRV values [32], 6 of 20 studies reported normalized units without raw values.

#### 3.4.3. Interpretation of HF, LF, and LF : HF Ratio (Table 8)

ECM and SCM studies (*n* = 14) interpreted HF as reflecting parasympathetic nervous system (PNS) mediated by RSA (Respiratory Sinus Arrhythmia) (*n* = 7); *n* = 6 as PNS, and *n* = 1 as RSA. This mirrors the debate on LF interpretation as a mix of sympathetic and vagal, and baroreceptor activities [58], and the ECM and SCM studies (*n* = 14) showed a mixed interpretation: baroreceptor activity (*n* = 1), more SNS than PNS (*n* = 5), baroreceptor + PNS (*n* = 1), baroreceptor + SNS + PNS (*n* = 3), SNS + balance of PNS and SNS (*n* = 1), and index of SNS (*n* = 3). Although all the ECM and SCM studies reported LF : HF as an index of sympathovagal balance, a recent consensus suggested lowering its predictive value [58], due to the loose relationship of LF power with sympathetic outflow [32], and the nonlinear and nonreciprocal relationship between SNS and PNS activity [59]. The discrepancy in HRV interpretation is problematic in deriving a conclusive insight on the correlation between constitutions and HRV.

The article "Exploring Heart Rate Variability as a Biomedical Diagnostic Tool for the Disympathetic Dimension of Eight-Constitution Medicine" was published in 2021. Journal: Evid Based Complement Alternat Med.

#### 3.4.4. Extraneous Factors Controlled for HRV (Table 9)

In general, some population variables (i.e., age, health condition, and medication) of ECM and SCM studies (*n* = 20) were well controlled (*n* = 14), but gender (*n* = 9) was relatively less controlled. Several procedure- and environment-related variables were frequently controlled (i.e., posture, resting, circadian rhythm, caffeinated drinks, alcohol, room lighting, or noise), with others less frequently controlled (i.e., smoking, wakefulness or talk, food, physical exercise, and temperature), and some not at all (i.e., bladder filling and stress level).

### 3.5. Classification of Constitutions

An ECM study [33] used pulse diagnosis with an intrarater reliability test (Kappa index 0.83%). SCM studies used QSCCII (Questionnaire for Sasang Constitution Classification) (*n* = 9), practitioner diagnosis based on SCAT (i.e., Sasang Constitution Analysis Tool including facial, voice, body, and QSCCII) (*n* = 6), practitioner diagnosis based on QSCCII (*n* = 4), and practitioner only diagnosis (*n* = 2).

## 4. Discussion

This systematic review explored HRV as a biomedical diagnostic for the Disympathetic Dimension of ECM.

### 4.1. Limitations of the Study

There are limitations to this review. The focus was on a qualitative and descriptive analysis of ECM and SCM studies on HRV reporting, interpretation, and control of extraneous factors. A review of statistical analysis including study population and effect size calculation was not within the study scope. Most articles were derived from the Korean research literature; despite the care with translation, misinterpretation or misunderstanding of the study contents is possible.

The article "Exploring Heart Rate Variability as a Biomedical Diagnostic Tool for the Disympathetic Dimension of Eight-Constitution Medicine" was published in 2021. Journal: Evid Based Complement Alternat Med.

### 4.2. Correlation between HRV and Constitution

The results of the systematic review showed little consistency in the data to support the use of HRV as an objective determinant of ECM constitutions.

1. A single ECM study of HRV differences after eight-constitution acupuncture had several limitations: sample size, control of age, and gender factors, and the data was not sufficient to draw meaningful conclusions on the use of HRV for constitutional differentiation along the Disympathetic Dimension
2. While consensus exists for HF as a proxy to evaluate cardiac vagal modulation when the respiratory frequency is mediated, LF and the LF/HF ratio lack a clear relationship to cardiac sympathetic modulation. None of the ECM and SCM studies reported significant differences between constitutions when measuring HF at resting. Two SCM studies showed some constitutional differences in the LF/HF ratio; however, the ratio lacks consensus as a reliable measure for sympathovagal balance [29, 30, 56]. The results alone, therefore, are not enough to explain the constitutional differences in terms of cardiac autonomic modulation.
3. While constitutional differences in HRV measures (i.e., SDNN, HFnu, LFnu, and LF/HF) in the SCM acupuncture stimulation studies are notable, there were limitations: HRV time domain values such as SDNN [21] are preferably computed through long-term recording (24 hours); therefore, the study result based on 30 seconds of SDNN requires further validation of reproducibility; LF/HF and LFnu are not sufficient to reflect cardiac autonomic modulation and changes in those measures alone have limited predictive value of constitutional differences.
4. While 5 out of 7 SCM acupuncture studies reported some HRV differences (HFnu, LFnu, LF/HF, and SDNN), the variety of study methods and procedure design made it difficult to compare, consolidate, and draw a robust conclusion. This variety includes: reporting of HRV measures (e.g., HFnu, LFnu, LF/HF, SDNN, and rMSSD), acupuncture methods and points (e.g., Taegeuk acupuncture, bee venom acupuncture, electroacupuncture at ST36 and ST38, acupuncture at LI4 or LI4 and LR3), frequency and duration (e.g., one session vs. three sessions over two weeks, 5 min vs. 15 min acupuncture), stimulation methods (e.g., only acupuncture vs. mental stress and acupuncture), study population (e.g., age, gender), HRV measurement timing (e.g., right after needle removal, 1 hour after needle removal), and control of extraneous factors (e.g., wakefulness or talk, food).

### 4.3. HRV Reporting and Interpretation

HRV reporting in the studies showed some opportunities to improve: inconsistency in the selection of HRV reporting measures, redundancy or inconsistent outcomes of normalized unit reporting (i.e., HFnu, LFnu, and LF/HF ratio) without raw values, and discrepancy in HRV interpretation (HF, LF, and LF/HF ratio). ECM and SCM studies reported only some of the HRV measures (i.e., mRR, SDNN, rMSSD, LF power, HF power, LFnu, HFnu, and LF : HF) that were recommended by a task force [58, 59] and the selection of measures were also inconsistent among the studies.

The article "Exploring Heart Rate Variability as a Biomedical Diagnostic Tool for the Disympathetic Dimension of Eight-Constitution Medicine" was published in 2021. Journal: Evid Based Complement Alternat Med.

### 4.4. Extraneous Factors

Among the HRV extraneous factors, some of the population variables (i.e., age, health condition, and medication) were well controlled, but gender and other procedural variables (e.g., wakefulness or talk, food) were less controlled in the studies.

In the studies examined, there was no clear relationship between HRV and Korean Constitutional Medicine, including the Disympathetic Dimension of ECM. Reasons included demographic discrepancies (i.e., age, gender, and health conditions), HRV reporting, methodological inconsistencies between the SCM studies, and insufficient ECM research. The continuing debates on whether HRV measures reflect autonomic function accurately add further complications on top of HRV's sensitivity to various extraneous factors.

## 5. Conclusions

This review examined HRV in the hope that it would be a useful objective diagnostic tool to bridge the information gap for acupuncture and traditional medicine researchers and, specifically, for determining a patient's position on the Disympathetic Dimension of Eight-Constitution Medicine. HRV does not seem to be suitable for this purpose alone.

## Figures and Tables

**Figure 1:** Eight constitutions and Disympathetic Dimension [5].

**Figure 2:** Systematic review process.

**Table 1:** Summary of studies investigating the correlation between Heart Rate Variability and Korean Constitution Medicine (ECM or SCM).

Reference	No.	Medicine	Population (age range)	Autonomic stimulus	Duration and HRV measures	Other measures
[33]	1	ECM	42 patients (14–73)	Eight-constitution acupuncture	5 min, frequency domain	BMI
[34]	2	SCM	32 healthy students (20–30)	Paced breathing in specific respiration rate	5 min, time and frequency domain	Respiration rate
[35]	3	SCM	60 healthy students (20–30)	Ratio of inhalation and exhalation, posture (sitting, standing)	Time and frequency domain	Self-evaluation for physical condition (scale 10 cm)
[36]	4	SCM	78 healthy students (20–30)	Breath-counting meditation	5 min, time and frequency domain	Skin conductance, temperature, abdominal amplitude, thoracic amplitude
[37]	5	SCM	78 students	Meditation program (*α* version)	Time and frequency domain	BDI (depression), STAXI (anger), STAI (anxiety) questionnaires
[38]	6	SCM	16 healthy TE constitution (20–60)	Taegeuk acupuncture	5 min, frequency domain	None
[39]	7	SCM	6 healthy SE constitution men (20–30)	Taegeuk acupuncture	5 min, frequency domain	None
[40]	8	SCM	63 fatigue and nonfatigue subjects (40–60)	None	5 min, time and frequency domain	BMI, biochemistry analysis, pulse wave analysis, nail fold capillary microscopy, questionnaires (FSS, GSRS, SF-MPQ, PSQI, SF-12)
[41]	9	SCM	8 healthy SY constitution women (20–30)	Taegeuk acupuncture	5 min, frequency domain	None
[42]	10	SCM	47 healthy subjects (29–66)	Forrest healing program (aroma, foods, tea by constitution + trekking)	5 min, time and frequency domain	BMI, body temperature, vital sign (BP, SpO2), electroencephalography, biochemistry analysis, blood cell count, stress hormone test
[43]	11	SCM	665 subjects (39–72)	None	5 min, time and frequency domain	BMI, BP, fasting blood sugar, cholesterol, abdominal obesity
[44]	12	SCM	20 healthy subjects (18–30)	Bee venom acupuncture	5 min, time and frequency domain	Pulse wave analysis, cerebral blood flow
[45]	13	SCM	103 idiopathic facial palsy patients (10–79)	None	5 min, time and frequency domain	Facial electromyography
[46]	14	SCM	10 TE constitution patients	Herbal formula for TE constitution (Jowisengcheong-tang)	5 min, time and frequency domain	None
[47]	15	SCM	30 healthy men (20–26)	Acupuncture at LI4	5 min, time and frequency domain	None
[48]	16	SCM	39 patients (20–59)	Autogenic training	5 min, time and frequency domain	MBTI questionnaire (extraversion, introversion)
[49]	17	SCM	8498 workers	None	5 min, time and frequency domain	None
[50]	18	SCM	44 healthy subjects (20–30)	Emotional stimulus (horror film)	120 sec, 197 sec, 120 sec, time and frequency domain	None
[51]	19	SCM	86 subjects (22–25)	Electroacupuncture	30 sec, time domain (SDNN)	None
[52]	20	SCM	19 healthy subjects	Acupuncture at LI4 and LR3	5 min, time and frequency domain	BP, BMI

ECM, Eight-Constitution Medicine; SCM, Sasang Constitution Medicine; CM, Constitution Medicine; HRV, Heart Rate Variability; MHR, mean heart rate; BMI, body mass index; TE, Taeumin constitution; SY, Soyangin constitution; FSS, Fatigue Severity Scale; GSRS, Gastrointestinal Symptom Rating Scale; SF-MPQ, Short-Form McGill Pain Questionnaire; PSQI, Pittsburgh Sleep Quality Index; SF-12, Short-Form Health Survey; BP, blood pressure; SpO_2_, peripheral capillary oxygen saturation; APG, Accelerated Plethysmogram; MBTI, Myers–Briggs Type Indicator.

The article "Exploring Heart Rate Variability as a Biomedical Diagnostic Tool for the Disympathetic Dimension of Eight-Constitution Medicine" was published in 2021. Journal: Evid Based Complement Alternat Med.

**Table 2:** HRV difference by constitution (*p* < 0.05), before and after acupuncture stimulation.

Reference	1 [33]	6 [38]	9 [41]	7 [39]	12 [44]	15 [47]	19 [51]	20 [52]
Constitution	ECM	SCM	SCM	SCM	SCM	SCM	SCM	SCM
Population (range)	42 patients (14–73)	16 healthy TE constitution (20–60)	8 healthy SY constitution women (20–30)	6 healthy SE constitution men (20–30)	20 healthy subjects (18–30)	30 healthy men (20–26)	86 subjects (22–25)	19 healthy subjects
Subjects by constitution group	Sympathicotonia = 22 (Pul, Col, Ren, Ves) Vagotonia = 20 (Hep, Cho, Pan, Gas)	TE = 16	SY = 8	SE = 6	SY = 5, TE = 8, SE = 7, TY = 0	SY = 8, TE = 13, SE = 9, TY = 0	SY = 34, TE = 27, SE = 25, TY = 0	SY = 6, TE = 7, SE = 6, TY = 0
Age and gender controlled by constitution group	na	na	Age, gender	Age, gender	Age	Age, gender	Age, gender	Age, gender
Acupuncture	Eight-constitution acupuncture	Taegeuk acupuncture (TE)	Taegeuk acupuncture (SY)	Taegeuk acupuncture (SE)	Bee venom acupuncture	Acupuncture at LI4	Electroacupuncture	Acupuncture at LI4 and LR3
HRV baseline difference by constitution	No difference	NA	NA	NA	No difference	Low in TE (LF/HF)	na	No difference

HRV by constitution compared to baseline, after acupuncture								
MHR	No difference	na	na	na	na	No difference	na	TE > SY, SE
mRR (ms)	na	na	na	na	na	na	na	
SDNN (ms)	na	na	na	na	No difference	No difference	SY > TE (passive)	TE > SY (active) SY > SE (general)
rMSSD (ms)	na	na	na	na	No difference	na	na	SE > TE^*∗*^
LF (ms^2^)	na	na	na	No difference	No difference	No difference	na	
HF (ms^2^)	na	na	na	No difference	No difference	No difference	na	
LFnu	na	Decreased in TE	Decreased in SY	No difference	na	Increased in SY	na	TE > SE^*∗*^
HFnu	na	Increased in TE	Increased in SY	No difference	na	na	na	SE, SY > TE^*∗*^
Ln (LF)	No difference	na	na	na	na	na	na	
Ln (HF)	No difference	na	na	na	na	na	na	
LF/HF	No difference	na	na	No difference	No difference	Increased in SY		
SE > SY	na	TE > SE^*∗*^						

ECM, Eight-Constitution Medicine; SCM, Sasang Constitution Medicine; Pul, Pulmotonia constitution; Col, Colonotonia constitution; Ren, Renotonia constitution; Ves, Vesicotonia constitution; Hep, Hepatonia constitution; Cho, Cholecystonia constitution; Pan, Pancreotonia constitution; Gas, Gastrotonia constitution; TE, Taeumin constitution; SY, Soyangin constitution; SE, Soeumin constitution; TY, Taeyangin constitution; MHR, Mean Heart Rate; na, not available; NA, not applicable.*∗*Compared to right after needle insertion vs. 1 hour after needle removal.

**Table 3:** HRV difference by constitution (*p* < 0.05), at resting.

Reference	8 [40]	11 [43]^1^	13 [45]	17 [53]^2^	15 [47]
Constitution	SCM	SCM	SCM	SCM	SCM
Population (age)	63 fatigue and nonfatigue subjects (40–60)	665 subjects (39–72)	103 idiopathic facial palsy patients (10–79)	8498 workers	30 healthy men (20–26)
Subjects by constitution group	Fatigue:	Total:	SY = 25 (M 7, F 18)	SY 4270	SY = 8, TE = 13,
	SY = 10, TE = 8,	SY = 100, TE = 363,	TE = 54 (M 27, F27)	TE 2331	SE = 9, TY = 0
	SE = 14, TY = 0	SE = 202, TY = 0	SE = 24 (M 8, F 16)	SE 1897	
	Nonfatigue:	Female <60 yrs	TY (0)	TY (0)	
	SY = 15, TE = 7,	SY = 36, TE = 140,			
	SE = 9, TY = 0	SE = 68, TY = 0			
Age and gender controlled by constitution group	Age	Age, gender (female < 60 yrs)	na	Gender	Age, gender
Type of study	Cross-sectional study (2012)	Cross-sectional study (Genomic cohort 2006)	Medical record retrospective review (2008–2009)	Health examination 2005	Acupuncture at LI4
MHR	na	No difference	No difference	No difference	No difference
mRR (ms)	na	na	na	na	na
SDNN (ms)	No difference	No difference	No difference	SE > TE	No difference
rMSSD (ms)	No difference	na	na	na	na
LF (ms^2^)	No difference	na	No difference	na	No difference
HF (ms^2^)	No difference	na	No difference	na	No difference
LFnu	No difference	SY > TE (all) SY > TE, SE (female, below 60 years)	na	na	na
HFnu	No difference	TE > SY (all) TE, SE > SY (female, below 60 years)	na	na	na
Ln (LF)	na	No	na	na	na
Ln (HF)	na	No	na	na	na
LF/HF	No difference	SY > TESY > TE, SE (female, below 60 years)	SY, TE > SE	No difference	Low in TE

SY, Soyangin constitution; TE, Taeumin constitution; SE, Soeumin constitution; M, male; F, female; na, not available. ^1^Multivariated adjusted odds ratio HRV analysis. The odds ratio adjusted for age, gender, education period, marital status, drinking status, smoking status, past history (hypertension, diabetes mellitus, and hyperlipidemia), BMI, and metabolic syndrome. ^2^HRV reporting generated indices (stress index, fatigue index) and TP showed a significant difference between constitution groups.

The article "Exploring Heart Rate Variability as a Biomedical Diagnostic Tool for the Disympathetic Dimension of Eight-Constitution Medicine" was published in 2021. Journal: Evid Based Complement Alternat Med.

**Table 4:** HRV difference by constitution (*p* < 0.05), controlled breathing.

Reference	4 [36]	2 [34]	3 [35]
Constitution	SCM	SCM	SCM
Population (age)	78 healthy students (20–30)	32 healthy students (20–30)	60 healthy students (20–30)
Subjects by constitution group	SY = 13, TE = 30, SE = 35, TY = 0	SY = 10, TE = 11, SE = 11, TY = 0	SY = 18, TE = 18, SE = 24, TY = 0
Age and gender controlled by constitution group	Age	Age	Age
HRV baseline difference by constitution	MHR : SY, SE > TE	No difference	No difference
HRV by constitution compared to baseline, with paced breathing	Breath-counting on inspiration and expiration (not controlling)	Paced breathing: 12, 6, or 3 times per min	Ratio of inhalation and exhalation (4 : 6, 6 : 4)
MHR	CIB : SE > TECEB : SE, SY > TE	No difference	No difference
mRR (ms)	na	No difference	No difference
SDNN (ms)	No difference	No difference	No difference
rMSSD (ms)	na	No difference	No difference
LF (ms^2^)	No difference	na	No difference
HF (ms^2^)	No difference	na	No difference
LFnu	na	na	No difference
HFnu	na	na	No difference
Ln (LF)	na	No difference	na
Ln (HF)	na	No difference	na
LF/HF	No difference	na	na

na, not available; CIB, Counting on Inspiration; CEB, Counting on Expiration.

The article "Exploring Heart Rate Variability as a Biomedical Diagnostic Tool for the Disympathetic Dimension of Eight-Constitution Medicine" was published in 2021. Journal: Evid Based Complement Alternat Med.

**Table 5:** HRV difference by constitution (*p* < 0.05), associated with other interventions.

Reference	5 [37]	10 [42]	14 [46]	16 [48]	18 [50]
Constitution	SCM	SCM	SCM	SCM	**SCM**
Population	78 students	47 healthy subjects (29–66)	10 TE patients	39 patients (20–59)	**44 healthy subjects (20–30)**
Subjects by constitution group	na	M (SY = 10, TE = 17, SE = 20, TY = 0) F (SY = 8, TE = 9, SE = 12, TY = 0)	TE = 10	SY = 9, TE = 12, SE = 18, TY = 0	**SY** **=** **10, TE** **=** **20 SE** **=** **14, TY** **=** **0**
Age and gender controlled by constitution group	na	Gender, age	na	na	**Age**
Intervention	Meditation program (*α* version)	Forrest healing program (aroma, foods, tea, trekking)	TE herbal formula (Jowisengcheong-tang)	Autogenic training	**Emotional stimulus (horror film)**
HRV baseline difference by constitution	No difference	No difference	na	No difference	**No difference**

HRV by constitution compared to baseline, associated with other interventions					
MHR	Decreased in SE Decreased in SY	Increased in SY	na	Decreased in TE	**na**
mRR (ms)	na	na	No difference	na	**No difference**
SDNN (ms)	Increased in SE	Decreased in SY	No difference	Increased in SE Increased in TE	No difference
rMSSD (ms)	Increased in SE	No difference	No difference	na	**na**
LF (ms^2^)	No difference	No difference	No difference	Na	**TE** **>** **SY, SE**
HF (ms^2^)	No difference	No difference	No difference	na	**No difference**
LFnu	No difference	No difference	No difference	No difference	**No difference**
HFnu	No difference	No difference	No difference	No difference	**No difference**
Ln (LF)	na	na	na	na	**na**
Ln (HF)	na	na	na	na	**na**
LF/HF	No difference	No difference	na	No difference	**No difference**

na, not available; M, male; F, female; SE, Soeumin constitution; SY, Soyangin constitution; TE, Taeumin constitution.

**Table 6:** Measures of short-term HRV reporting (20 studies).

	HRV measures	1	2	3	4	5	6	7	8	9	10	11	12	13	14	15	16	17^*∗∗*^, *∗*	18	19	20	Total
Time domain	mRR (ms)^*∗*^		✓	✓											✓				✓			4
	**SDNN (ms)** ^*∗*^		✓	✓	✓	✓			✓		✓	✓	NR	✓	✓	✓	✓	✓	✓	✓	✓	16
	rMSSD (ms)^*∗*^		✓	✓		✓			✓		✓		NR		✓						✓	8

Frequency domain	**LF (ms** ^**2**^ **)** ^*∗*^			✓	✓	✓		✓	✓		✓		NR	✓	✓	✓	✓		✓			12
	**HF (ms** ^**2**^ **)** ^*∗*^			✓	✓	✓		✓	✓		✓		NR	✓	✓	✓	✓		✓			12
	LFnu^*∗*^			✓		✓	✓	✓	✓	✓	✓	✓			✓				✓		✓	11
	HFnu^*∗*^			✓		✓	✓	✓	✓	✓	✓	✓			✓				✓		✓	11
	**LF:HF** ^*∗*^	✓			✓	✓		✓	✓		✓	✓	NR	✓	✓	✓	✓	✓			✓	14
																					
	ln (LF)	✓	✓									✓										3
	ln (HF)	✓	✓									✓										3

Other measures	MHR (bpm)	✓	✓	✓	✓	✓					✓	✓		✓		✓	✓	✓	✓		✓	13
	MRR (BPM)		✓																			1
	BP (mmHG)										✓	✓									✓	3

Single vs. multiple Nu/ratio		M	M	M	S	M	M	M	M	M	M	M	S	S	M	S	S	S	M	na	M	

Raw (Y, N)		n	n	y	y	y	n	y	y	n	y	y	y	y	y	y	y	n	y	na	n	

NR = not reported; na, not applicable; mRR = mean RR interval; SDNN = standard deviation of normal-to-normal intervals; rMSSD = root mean square of successive differences; LF = low-frequency spectral power; HF = high-frequency spectral power; LF : HF = ratio of low-frequency power to high-frequency power; nu = normalized units; ln = natural logarithm; MHR = mean heart rate; MRR = mean respiration rate; BP = blood pressure. ^*∗*^The approved task force measures of short-term HRV [56,57]; ^*∗∗*^, *∗*indices from HRV device (nonstandard measures, e.g., stress index and fatigue index).

The article "Exploring Heart Rate Variability as a Biomedical Diagnostic Tool for the Disympathetic Dimension of Eight-Constitution Medicine" was published in 2021. Journal: Evid Based Complement Alternat Med.

**Table 7:** Reporting raw vs. adjusted values and single vs. multiple normalized ratio units^*∗*^.

	Raw values	No raw values	
Single nu/ratio unit	5	1	6
Multiple nu/ratio unit	8	5	13
	13	6	*n* = 19

^*∗*^Table format [32].

**Table 8:** Various explanations given as the sources of the short-term HRV measures (20 studies).

HRV measures	Explanations	1	2	3	4	5	6	7	8^*∗*^	9	10	11	12^*∗*^	13	14^*∗*^	15	16	17	18^*∗*^	19^+^	20	Total	
Year		2005	2016	2016	2015	2014	2013	2013	2013	2012	2011	2009	2009	2009	2008	2007	2007	2007	2007	2006	2004		

LF	SNS						✓										✓				✓	3	14
	SNS > PNS				✓	✓		✓		✓						✓						5	
	SNS, BAL											✓										1	
	BAR, SNS, PNS	✓									✓							✓				3	
	BAR, PNS		✓																			1	
	BAR			✓																		1	

HF	RSA, PNS	✓	✓		✓					✓	✓	✓				✓						7	14
	PNS					✓	✓	✓									✓	✓			✓	6	
	RSA			✓																		1	

LF : HF	BAL	✓						✓		✓	✓	✓		✓		✓	✓	✓			✓	10	10

BAR, the activity of Baroreflex; PNS, parasympathetic nervous system; SNS, sympathetic nervous system; RSA, respiratory sinus arrhythmia; BAL, a balance of sympathetic and parasympathetic influences. ^*∗*^Explanation on HRV measures not reported; ^+^not applicable.

**Table 9:** Extraneous factors controlled for HRV (20 studies).

	Extraneous factors	1	2	3	4	5^*∗*^	6	7	8	9	10^*∗*^	11^*∗*^	12	13	14	15	16	17	18	19	20	Total
Study population	Age		✓	✓	✓			✓	✓	✓	✓	✓	✓			✓			✓	✓	✓	13
	Gender							✓		✓	✓	✓				✓		✓		✓		7
	Health condition	✓	✓	✓	✓		✓	✓	✓	✓^*∗∗*^		✓	✓		✓	✓	✓		✓	✓	✓	16
	Medication	✓	✓	✓	✓		✓	✓	✓	✓		✓	✓		✓	✓	✓		✓		✓	15
	BMI	✓									✓	✓									✓	4

Sample size		42	32	60	78	78	16	6	63	8	47	665	20	103	10	30	39	8498	44	86	19	

Study procedure	Posture	✓^1^	✓^1^	✓^2^	✓^3^		✓^1^	✓^1^	✓^1^	✓^1^		✓^3^	✓^1^	✓^1^	✓^1^	✓^1^	✓^3^			✓^1^	✓	16
	Resting	✓^a^	✓^b^	NA	NA		✓^b^	✓ ^b^	✓ ^b^	✓ ^b^			✓ ^b^	✓ ^b^	✓ ^c^	✓ ^a^	✓^d^		✓ ^a^	✓^b^		13
	Circadian rhythm		✓	✓	✓		✓	✓		✓			✓		✓	✓					✓	10
	Wakefulness, talk			✓	✓											✓	✓		✓	✓	✓	7
	Caffeinated drinks	✓	✓	✓	✓		✓	✓		✓				✓		✓	✓					10
	Alcohol	✓	✓	✓	✓		✓	✓		✓				✓		✓	✓					10
	Smoking	✓					✓	✓		✓				✓		✓	✓					7
	Food	✓		✓			✓	✓		✓						✓						6
	Bladder filling																					0
	Physical exercise						✓	✓		✓												3
	Stress level																					0

Study environment	Light	✓					✓	✓	✓	✓			✓		✓				✓	✓		9
	Noise	✓	✓	✓	✓		✓	✓	✓	✓			✓		✓	✓			✓	✓		13
	Temperature	✓																	✓			2

Factors total = 19		12	9	10	10	0	12	14	7	14	1	6	8	5	7	13	8	1	8	8	7	

NA, not applicable; ^a^10 min resting before HRV; ^b^5 min resting before HRV; ^c^resting time not available; ^d^1 min resting before HRV; ^1^supine; ^2^sitting and standing; ^3^sitting; ^*∗*^information on HRV control factors not available; ^*∗∗*^menstruation factor controlled; ^+^multivariated adjusted odds ratio analysis (age, gender, BMI, alcohol drinking status, smoking status, health condition, metabolic syndrome, marital status, and education level); 9 am to 4 pm (wide range).

The article "Exploring Heart Rate Variability as a Biomedical Diagnostic Tool for the Disympathetic Dimension of Eight-Constitution Medicine" was published in 2021. Journal: Evid Based Complement Alternat Med.

## Data Availability

The datasets used and analyzed during the current study are available from the corresponding author on reasonable request.

## Abbreviations

ECG: Electrocardiogram
ECM: Eight-constitution medicine
HF: High frequency
HFnu: Normalized high frequency
HRV: Heart rate variability
IBI: Interbeat intervals
KCM: Korean constitution medicine
LF: Low frequency
LFnu: Normalized low frequency
LI4: Large intestine 4
LR3: Liver 3
mRR: Mean of R-R intervals
SCM: Sasang constitution medicine
SDNN: Standard deviation of NN intervals
PPG: Photoplethysmogram
rMSSD: Root mean square of the successive differences.
